# Endothelial Dysfunction, Inflammation, and Oxidative Stress in COVID-19—Mechanisms and Therapeutic Targets

**DOI:** 10.1155/2021/8671713

**Published:** 2021-08-21

**Authors:** Adriana Fodor, Brandusa Tiperciuc, Cezar Login, Olga H. Orasan, Andrada L. Lazar, Cristina Buchman, Patricia Hanghicel, Adela Sitar-Taut, Ramona Suharoschi, Romana Vulturar, Angela Cozma

**Affiliations:** ^1^Clinical Center of Diabetes, Nutrition, and Metabolic Diseases, “Iuliu Haţieganu” University of Medicine and Pharmacy, 400012 Cluj-Napoca, CJ, Romania; ^2^Department of Pharmaceutical Chemistry, “Iuliu Haţieganu” University of Medicine and Pharmacy, 400012 Cluj-Napoca, Romania; ^3^Department of Physiology, “Iuliu Haţieganu” University of Medicine and Pharmacy, 400012 Cluj-Napoca, CJ, Romania; ^4^Internal Medicine Department, 4th Medical Clinic “Iuliu Haţieganu” University of Medicine and Pharmacy, 400012 Cluj-Napoca, Romania; ^5^Department of Dermatology, “Iuliu Haţieganu” University of Medicine and Pharmacy, 400006 Cluj-Napoca, Romania; ^6^Department of Oncology, “Iuliu Haţieganu” University of Medicine and Pharmacy, 400015 Cluj-Napoca, Romania; ^7^Department of Neurology, “Iuliu Haţieganu” University of Medicine and Pharmacy, 400012 Cluj-Napoca, Romania; ^8^Department of Food Science, University of Agricultural Science and Veterinary Medicine, 400372 Cluj-Napoca, Romania; ^9^Department of Molecular Sciences, “Iuliu Haţieganu” University of Medicine and Pharmacy, 400012 Cluj-Napoca, Romania

## Abstract

The outbreak of the COVID-19 pandemic represents an ongoing healthcare emergency responsible for more than 3.4 million deaths worldwide. COVID-19 is the disease caused by SARS-CoV-2, a virus that targets not only the lungs but also the cardiovascular system. COVID-19 can manifest with a wide range of clinical manifestations, from mild symptoms to severe forms of the disease, characterized by respiratory failure due to severe alveolar damage. Several studies investigated the underlying mechanisms of the severe lung damage associated with SARS-CoV-2 infection and revealed that the respiratory failure associated with COVID-19 is the consequence not only of acute respiratory distress syndrome but also of macro- and microvascular involvement. New observations show that COVID-19 is an endothelial disease, and the consequent endotheliopathy is responsible for inflammation, cytokine storm, oxidative stress, and coagulopathy. In this review, we show the central role of endothelial dysfunction, inflammation, and oxidative stress in the COVID-19 pathogenesis and present the therapeutic targets deriving from this endotheliopathy.

## 1. Introduction

The SARS-CoV-2 virus, responsible for COVID-19 disease, can evolve with a wide range of clinical manifestations, from mild forms manifesting as fever, dyspnea, cough, and loss of smell and taste to severe forms, especially in the elderly with comorbidities, characterized by respiratory failure due to severe alveolar damage [1]. In the extremely severe forms of the disease, rapidly progressive multiple organ failure occurs, which manifests through complications such as shock, acute cardiac injury, acute respiratory distress syndrome (ARDS), disseminated intravascular coagulopathy (DIC), and acute kidney injury, which may ultimately prove fatal [2]. Recent studies have demonstrated that respiratory failure occurring in COVID-19 is due not only to acute respiratory distress syndrome but also to macro- and microvascular involvement [3–5], a particular role being played by vascular endothelial damage [6, 7]. New observations show that COVID-19 is an endothelial disease [8] and that endotheliopathy is responsible for inflammation, cytokine storm, oxidative stress, and coagulopathy. An argument of this theory is the fact that patients who have endothelial dysfunction due to various comorbidities (obesity, hypertension, and diabetes) develop more severe forms of COVID-19, explained by an additional alteration of the already dysfunctional vascular endothelium [7].

In this review, we show the central role of endothelial dysfunction, inflammation, and oxidative stress in the development of complications of SARS-CoV-2 infection and their pathophysiological consequences, and examine the main therapeutic targets deriving from this endotheliopathy.

The endothelium, one of the largest organs of the human body, is capable of producing a wide variety of molecules, with effects that are often contradictory, with a role in maintaining homeostasis, such as vasodilator and vasoconstrictor, procoagulant and anticoagulant, inflammatory and anti-inflammatory, fibrinolytic and antifibrinolytic, and oxidant and antioxidant substances [9].

The normal endothelium regulates vascular homeostasis through six major functions: (1) modulation of vascular permeability, (2) modulation of vasomotor tone, (3) modulation of coagulation homeostasis, (4) regulation of inflammation and immunity, (5) regulation of cell growth, and (6) oxidation of LDL cholesterol (Figure 1). These functions are achieved through numerous mediators, of which the most studied is nitric oxide (NO) [9].

Nitric oxide is the most important vasodilator substance produced by endothelial cells. NO also has an antithrombotic action, inhibiting the fibrotic properties of angiotensin II and endothelin I by downregulating the receptors for these molecules. NO is synthesized in endothelial cells from L-arginin under the action of the endothelial NO synthase (eNOS) [10]. This reaction requires the presence of molecular oxygen and certain cofactors, including calmodulin, tetrahydrobiopterin (THB4), NADPH (adenine dinucleotide phosphate), flavin adenine dinucleotide, and flavin mononucleotide. From this reaction, L-citrulline as a by-product results [11].

Endothelial dysfunction is defined as a reduction in the bioavailability of vasodilator substances, especially NO, and an increase in vasoconstrictor substances.

The reduction of NO bioavailability can be due to a decrease in eNOS production (lack of cofactors necessary for eNOS synthesis) on the one hand, and to an increase in excessive NO degradation or inactivation by reactive oxygen species (ROS), on the other hand [12]. The increase in the production of ROS, such as superoxide anion (O_2_^−^), hydrogen peroxide (H_2_O_2_), hydroxyl radical (HO^•^), hypochlorous acid (HOCl), and lipid superoxide radical, represents the main cause of the decrease in NO bioavailability in cardiovascular diseases [13]. Under physiological conditions, ROS production is controlled by an effective system of antioxidants, molecules that are capable of neutralizing ROS, thus preventing oxidative stress. In tissues, natural enzymatic antioxidants, such as superoxide dismutase (SOD), glutathione peroxidase, and catalase, play an important role in the conversion of ROS to oxygen and water. In pathological conditions, ROS can be present in excess relatively to the existing antioxidant capacity. This alteration of the balance in favor of oxidation termed “oxidative stress” may have negative effects on cell and tissue function [9].

Endothelial cells (EC) possess a number of mechanisms that reduce local oxidative stress. When subjected to shear stress, the endothelium produces SOD, which eliminates ROS [14]. The endothelial cell can also express glutathione peroxidase, which can mitigate oxidative stress [15]. Similarly, haem-oxygenase provides another mechanism by which the endothelial cell can resist to local oxidative stress [16, 17].

In contrast, proinflammatory cytokines can stimulate endothelial cells to mobilize NADPH-oxidase that generates superoxide anions, amplifying local oxidative stress [18, 19].

## 2. COVID-19-Associated Endotheliopathy and Oxidative Stress

Endothelial dysfunction or endotheliopathy is an important pathological characteristic in COVID-19 [20]. Electron microscopy of blood vessels in autopsy samples from patients with COVID-19 revealed the presence of endothelial cell degradation and apoptosis [21, 22]. Endothelial dysfunction biomarkers, such as thrombomodulin, von Willebrand factor (vWF), angiopoietin 2, and PAI-1, are frequently increased in patients with COVID-19 compared to healthy persons and seem to have prognostic significance, being associated with more severe forms of the disease and high mortality [23, 24]. Endothelial dysfunction is an important factor in the pathophysiology of thrombotic complications associated with COVID-19, including myocardial infarction and stroke [23, 24].

At present, it is uncertain whether endotheliopathy associated with COVID-19 is the result of direct endothelial cell viral infection, as reported in some autopsy studies [21, 25] or is a consequence of the inflammatory response induced by the virus.

Many pathophysiological mechanisms have been described which explain the implication of endothelial dysfunction in the occurrence of microvascular involvement in COVID-19 infection. Microvascular cerebral involvement in COVID-19 as a result of age-related endothelial dysfunction is an important challenge for research [20]. Overactivation of poly-(ADP-ribose) polymerase 1, as can be observed in viral infections, can lead to NAD+ depletion and subsequent endothelial dysfunction [26, 27]. In addition, the dysfunction of the nuclear factor erythroid 2-related factor 2 (NRF2) antioxidant defense pathway in endothelial cells might also play a role in the COVID-19 associated endotheliopathy [28]. The pharmacological activators of NRF2 were proposed as potential treatment options for COVID-19 [29]. NRF2 has strong anti-inflammatory and antiapoptotic effects in endothelial cells. It should be noted that NRF2 dysfunction exacerbates the deleterious effect of hypertension and diabetes on the endothelium, conditions known for the increase in the COVID-19-related risk of death [29].

Oxidative stress is generated by high Ang II concentrations and low Ang 1-7 concentrations (Figure 2). These ROS can oxidize cysteine residues in the peptidase domain of receptors ACE2 and RBD of proteins SARS-CoV and SARS-CoV-2, maintaining them in oxidized forms (disulfide), unlike reduced forms (thiol) [30]. It is possible that oxidation of these thiols to disulfides, through an oxidative stress mechanism, may increase the affinity of proteins SARS-CoV and SARS-CoV-2 S for ACE2 receptors and, consequently, increase the severity of COVID-19 infection [31].

The relationship between Ang II and NADPH-oxidase was investigated using murine smooth vascular muscle cells. When the cells were exposed to Ang II, the researchers observed an increased activity of NADPH-oxidase, as well as an increased production of superoxide anions. The exact mechanisms for the stimulation of NADPH-oxidase are complex, genetically mediated, at transcriptional and posttranscriptional level, and involve numerous signaling molecules and scaffolding proteins/platforms [32]. Inactive NADPH-oxidase contains two subunits: glycoprotein (gp) 91phox and p22phox. In the presence of Ang II, NADPH-oxidase is activated through the involvement of additional subunits p67phox, p47phox, p40phox, and Rac1. Activated NADPH-oxidase can generate superoxide anions. Studies in mice have shown that increased NADPH-oxidase activity can be found even in the absence of ACE2 [33, 34]. Since binding of SARS-CoV-2 to ACE2 receptor inhibits the catalytic activity of the enzyme, i.e., the conversion of Ang II to Ang 1-7, the activity of NADPH-oxidase increases in patients with SARS-CoV-2, subsequently leading to an increase in oxidative stress [35].

In a recently published study [36], the long-term effects of SARS-CoV-2 virus on oxidative stress and vascular endothelium were discussed. Thus, it was proposed that SARS-CoV-2, by inducing mitochondrial dysfunction and oxidative stress, can initiate a feedback loop promoting a chronic state of inflammation and endothelial dysfunction even after the viral particles have been eliminated from the body. In this proposed mechanism, SARS-CoV-2 first induces activation of NADPH-oxidase, which produces superoxide (O_2_^–^), a ROS that is involved in reactions which deteriorate the electron transport chain (ETC) [32, 37].

Increased oxidative stress and inflammation resulting from this mitochondrial dysfunction subsequently initiate a feedback loop that perpetuates NADPH-oxidase activation, mitochondrial dysfunction, inflammatory cytokine production and loss of identity of EC [36]. Considering these hypothetical long-term consequences of SARS-CoV-2 infection on blood vessels, the treatment of chronic oxidative stress and inflammation in EC can be essential in preventing future complications among millions of persons currently diagnosed with COVID-19 [38].

## 3. COVID-19 Endotheliitis

Numerous postmortem histopathological examinations in patients who died of COVID-19 not only revealed the presence of endotheliitis in the key organs affected by SARS-CoV-2, but also demonstrated the presence of viral structures within the endothelial cells by electron microscopy [21, 25, 39, 40]. By analyzing samples from the transplanted kidney in a COVID-19 patient who developed multiorgan failure, Varga et al. [25] demonstrated the capacity of the virus to invade endothelial cells. In the same patient, histological findings showed the inflammatory infiltrate of the endothelium and the morphological changes that occur during apoptosis in the heart, small bowel, and lungs. Furthermore, they proved the presence of endotheliitis in the lung, heart, kidney, liver, and small intestine of two other COVID-19 patients by postmortem analysis [25]. The wide distribution of ACE2 receptor in endothelial cells explains the multiorgan affinity of the virus, confirmed once more in a study by Puelles et al. The presence of viral particles in the pharynx, lungs, heart, blood, liver, kidneys, and brain was established despite the level of viral load [39].

The electron microscopy studies performed by Ackermann et al. [21] proved the presence of SARS-CoV-2 within the endothelial cells and in the extracellular space; furthermore, ultrastructural injury of the endothelium was also present. The authors of the aforementioned study compared the histological changes that occur in the lungs of SARS-CoV-2 patients with those occurring in acute respiratory distress syndrome caused by influenza A (H1N1) and ten uninfected control lungs. The results revealed that the lungs of COVID-19 patients presented disseminated alveolar injury associated with necrosis, lymphocytic inflammation, and microthrombosis. In addition, the expression of angiotensin-converting enzyme 2 (ACE2) investigated by immunohistochemical analysis was present in lymphocytes only in the COVID-19 and influenza groups [21].

The postmortem electron microscopy analysis of the kidney tissue of 26 patients with COVID-19 from China revealed the presence of coronavirus-like particles in the renal tissue. Furthermore, the SARS-CoV-2 receptor ACE2 was upregulated in these patients. This study conducted by Su et al. confirms once more the virus tropism for kidney tissue [40].

Menter et al. identified in patients who died with COVID-19 the presence of capillaritis and microthrombi in the lungs, and showed diffuse vascular damage in other organs highly suggestive of vascular dysfunction [41].

Cutaneous biopsies from the skin lesions associated with SARS-CoV-2 were also performed. The optical microscopy findings of a biopsy from a chilblain-like lesion in a 23-year-old patient diagnosed with coronavirus disease revealed the presence of inflammatory infiltrate, consisting especially of lymphocytes, which were “tightly cuffing the vessels” [42]. Kanitakis et al. accomplished histological, immunofluorescence, and immunohistochemical studies in seventeen cases of acral chilblain-like skin lesions in patients with suspected, but not confirmed, coronavirus disease, and endotheliitis was present in 65% of cases [43]. The association of COVID-19 with chilblain-like skin lesions is still conflicting. Initially, acral lesions were thought to be related to SARS-CoV-2 infection, but more recent case studies could not sustain an association between them [43, 44].

All data collected from the autopsies indicate that changes in the endothelium are not limited to the lungs and suggest that COVID-19 is a whole-body disease.

Numerous symptoms of SARS-CoV-2-positive patients could be assigned to multiorgan endotheliitis and subsequent endothelial dysfunction.

As mentioned above, tropism for the kidneys, lungs, and cardiovascular system of the novel coronavirus was demonstrated. This explains the respiratory and cardiocirculatory events associated with the disease. Several hypotheses were proposed in order to explain other organ specific symptoms. The early neurological manifestations (hyposmia, anosmia, dysgeusia, or hypogeusia) which have been frequently described in these patients together with life threatening events such as stroke and intracerebral or subarachnoid hemorrhage could represent a consequence of endotheliitis [45]. In a short communication, Benger et al. made a detailed analysis of 5 patients with COVID-19 and intracerebral hemorrhage. They suggest that endothelial damage and endotheliitis along with a prothrombotic state and proinflammatory cytokine production are responsible for intracerebral hemorrhage, which occurred in younger individuals. Hemorrhage affected the anterior cerebral circulation [46].

In addition to the detrimental effect on blood vessels, the heart also represents a target for SARS-CoV-2. The main cardiovascular manifestations of COVID-19 are cardiac arrhythmias, caused by the inflammation of the myocardium and metabolic dysregulation [47]. It has been suggested that both direct and indirect viral injury is responsible for COVID-19-associated myocarditis [48].

The emerging evidence recognizes the endothelium as a key factor in the pathophysiological chain in COVID-19 [49]. Therefore, arterial and venous thrombosis, pulmonary embolism [49], central nervous system acute hemorrhagic events, and multiorgan failure associated with SARS-CoV-2 infection [50] might be the aftermath of subsequent endotheliitis and endothelial dysfunction associated with a procoagulant state. Endothelial cell damage together with endotheliitis also explains the predisposition for severe manifestations of the disease in patients with preexisting endothelial dysfunction caused by chronic pathologies such as hypertension [47].

While the major role of endothelial cells in the pathophysiology of COVID-19 is a compelling subject for ongoing research projects, the hypothesis according to which the endothelium could represent a therapeutic target in critically ill patients is intensely analyzed [49].

## 4. COVID-19-Renin-Angiotensin System

The role of the renin-angiotensin-aldosterone system (RAAS) in COVID-19 infection has been taken into consideration from the beginning of the pandemic, since one of the first known facts was that ACE2 (angiotensin-converting enzyme 2) is the receptor that allows SARS-CoV-2 to enter human cells.

RAAS is a natural protective mechanism for maintaining circulatory volume. Renal hypoperfusion stimulates renin release from the juxtaglomerular apparatus. Renin cleaves angiotensinogen to angiotensinogen I, and ACE hydrolyzes Ang I to Ang II. Ang II binds to angiotensin II type 1 receptor (AT1R) and promotes aldosterone production, leading to sodium retention, water reabsorption, and vasoconstriction. On the other arm of the cascade, ACE2 is maintaining the equilibrium by converting Ang II to angiotensin 1-7. Angiotensin 1-7 binds to the Mas receptor and mediates anti-inflammatory, antioxidative, and vasodilatory effects. In the case of insufficient ACE2, Ang II binding AT1R prevails and exerts vasoconstrictive and proinflammatory effects [51].

Angiotensin-converting enzyme 2 (ACE2) is expressed in the human vascular endothelium, respiratory epithelium, and other types of cells, and represents a primary mechanism for the entry and infection of SARS-CoV-2 virus. In a physiological state, ACE2 through the activity of carboxypeptidase generates angiotensin fragments (Ang 1-9 and Ang 1-7) and plays an essential role in the renin-angiotensin system (RAS), which is an important regulator of cardiovascular homeostasis. SARS-CoV-2 through its surface glycoprotein interacts with ACE2 and invades the host cells.

For SARS-CoV-2 infection, in addition to ACE2, one or more proteases including transmembrane protease serine 2 (TMPRSS2), basigin (also known as CD147), and potentially cathepsin B or cathepsin L are required [52].

ACE2 is expressed as a transmembrane protein whose active site is exposed at the extracellular surface and resides in the lung alveolar epithelial cells, heart, kidneys, vessels, and gastrointestinal system [53]. ACE2 can be cleaved and circulates in small amounts in the blood stream, but its role is uncertain [54–57].

While ACE2 is clearly responsible for facilitating cell insertion, it may also be the cause of individual variation in disease severity. The polymorphism of ACE2 in the population could impact the affinity for the virus's spike protein and make the infection more likely or more severe [57]. Also, the ACE2 gene is X-linked, and this could explain the slight protective effect in the female sex observed in COVID-19. Besides these genetic variations, ACE2 gene expression is increased in diabetes, CVD, and hypertension [58]. Several researches indicate that RAAS-modulating drugs could also modulate ACE2 expression and activity in various ways. Animal model studies have shown that ACE inhibitors (ACEIs) and angiotensin II receptor blockers (ARBs) upregulate ACE2 cell expression, and ARBs and mineralocorticoid receptor antagonists (MRA) increase ACE2 activity, [59, 60]. However, simultaneously, ACEIs reduce Ang II synthesis, and consequently, in the absence of excess Ang II, AT1R is thought to interact with ACE2 [61]. This interaction could reduce the affinity of COVID S protein to ACE2 and then reduce COVID-19 viral entry [61].

SARS-CoV-2 spike protein binding to ACE2 in alveolar epithelial cells downregulates ACE2 expression. Without ACE2 to lead Ang II to angiotensin 1-7, Ang II binds to AT1R, leading to a hyperaldosteronism state, materialized as hypokalemia in severe cases of COVID-19 infection [62], vasoconstriction, fibrosis, and inflammatory cell proliferation [63]. Murine studies proved that loss of ACE2 expression enhances vascular permeability, increases lung edema and neutrophil accumulation, and hence worsening lung function [64].

One of the earliest researches of Chinese scientists empowers the theory that excessive Ang II leads to a bad outcome. Liu et al. observed in a small cohort of COVID-19 patients that the plasma concentrations of Ang II were significantly higher than in healthy individuals and also that Ang II levels in COVID-19 patients were correlated with viral load and lung injury [65].

Besides exacerbated inflammation and hypoxemia through vasoconstriction in small pulmonary vessels, Ang II induces plasminogen activator inhibitor-1 (PAI-1) expression in endothelial cells via the AT1 receptor. PAI-1 leads to unresolved fibrin deposits in the alveoli of patients with both SARS and COVID-19 infection [51]. Also, excessive Ang II can be metabolized to angiotensin IV [66], which enhances thrombosis development [67, 68]; since hypercoagulability has been noticed in many severe cases, it can be hypothesized that a reduction in ACE2 contributes to increasing thrombotic risk.

Since ACE2 has been recognized as the gate of SARS-CoV-2, worldwide medical boards raised the question if RAAS modulators—ACEIs and ARBs—increase the risk of developing severe forms of COVID-19 infection. The rationale behind this concern was based on some experimental animal models which have shown increasing numbers of ACE2 after intravenous infusion of ACEIs and ARBs [59].

In order to establish whether RAAS modulators are harmful or not, scientists firstly compared the outcomes of COVID-19 patients with arterial hypertension and different treatments. Shyh et al. found that those on ARBs are significantly less likely to develop COVID-19, while ACEIs did not show a similar effect, considering that they do not directly affect ACE2 activity [69]. On the other hand, patients taking calcium channel-blockers (CCBs) had a significantly increased risk of manifesting symptoms of COVID-19.

Several other retrospective multicenter studies [63, 70] looked for an association between in-hospital use of ACEIs/ARBs and all-cause mortality of COVID-19 among patients with hypertension. Their results show that COVID-19 hypertensive patients treated with ACEIs/ARBs had a better outcome than COVID-19 patients without ACEIs/ARBs or treated with a different class of other antihypertensive agents. On a molecular basis, they identified that patients on ACEIs/ARBs had lower levels of IL-6, decreased cytokine production, and decreased viral load during hospitalization, and peripheral T cells were significantly higher than in the non-ACEI/ARB group [70].

Researchers' restless work not only offered substantial information about the role of ACE2 in COVID-19 infection, but also brought up several potential therapeutic approaches: spike protein-based vaccine, inhibition of transmembrane protease serine 2 (TMPRSS2-human proteinase which facilitates viral spike protein binding to ACE2) activity, blocking ACE2 receptor, and delivering an excessive soluble form of ACE2 [71]. It was postulated that delivering excessive soluble ACE2 would capture most of the viral load, restricting their fixation on cell membrane ACE2, and therefore limit the infection and also keep the balance of the 2 RAAS arms, preventing severe inflammatory tissue lesions [72, 73]. Most of these theories are based on animal model or in vitro studies and, needless to say, require extensive research and trials before becoming available therapies.

## 5. Cytokine Storm Associated with SARS-CoV-2 Infection

About 5% of the patients infected with SARS-CoV-2 develop critical disease forms manifesting by respiratory failure, shock, or multiple organ failure [74]. The presence of these disease forms does not seem to be correlated with viral load. Although these patients have a high viral load, the same load is found in patients having mild forms of the disease and even in asymptomatic persons [75]. Thus, the hypothesis was advanced that abnormal immune response, manifesting as a “cytokine storm,” is the main determining factor of disease severity [76].

Cytokine storm associated with COVID-19 is similar to other clinical entities, such as cytokine release syndrome observed following CAR-T cell therapy [77], primary or secondary hemophagocytic lymphohistiocytosis (HLH), sepsis caused by Herpesviridae and other pathogens [78], and macrophage activation syndrome that occurs in various autoimmune diseases [79].

This progressive systemic inflammation leads to the loss of vascular tone clinically manifesting by a decrease in blood pressure, vasodilatory shock, and progressive organ failure. In the context of cytokine storms associated with highly pathogenic viruses such as SARS-CoV-2, SARS-CoV, and MERS-CoV, the greatest impact is on the lungs, where acute respiratory distress syndrome (ARDS) occurs which is the main cause of death. The effects are not limited to the lungs; cardiac, renal, and central nervous system damage is also involved [80].

After receptor binding and complex internalization, the viral RNA is released into the cell cytosol, replicated, and finally removed by exocytosis.

Intracellular viral RNA is identified by the recognition mechanisms of the innate immune response through specific receptors: PRRs (pattern recognition receptors), TLRs (toll-like receptors), and NLRs (NOD-like receptors). The recognition of viral RNA by these receptors determines the activation of intracellular signaling pathways, such as NF-*κ*B and IRF 3/7. NF-*κ*B stimulates the transcription of proinflammatory cytokines such as TNF-alpha, IL-6, and IL-1 and activates the immune response mediated by T helper 1 and 17 lymphocytes. IRF 3/7 stimulates the production of type 1 IFN, which induces activation of the JAK1/TYK2-STAT1/2 pathway, the effect being the transcription of interferon-stimulated genes (ISG), with a role in the secretion of cytokines and the activation of other immune system components to stop viral replication [81, 82].

Previous studies have shown that in some cases, coronaviruses can delay type I IFN response through various mechanisms, the result being a more severe form of the disease caused by ineffective viral replication control and paradoxical hyperinflammation caused by type I IFN. In the case of SARS-CoV-2, an altered response of type I IFN seems to occur. A study showed that serum IFN activity was significantly lower in patients with severe or critical forms of the disease compared to those with mild-moderate forms. Moreover, serum ISG and type I IFN values in patients who subsequently developed ARDS with the need for invasive ventilation indicated that a mitigated type I IFN response precedes clinical deterioration [83].

This abnormal response of interferon leads to a massive inflow of neutrophils and monocytes, which are a major source of proinflammatory cytokines, apoptosis of T lymphocytes, and epithelial and endothelial cells [81].

Lymphopenia occurs in about 80% of the patients infected with SARS-CoV-2 and is more marked in the severe forms of the disease. There are many causal hypotheses explaining this process. Firstly, the virus can directly infect T lymphocytes but cannot replicate inside these, thus leading to cell death through apoptosis, necrosis, or pyroptosis. Secondly, the first wave of cytokines released, described above, includes anti-inflammatory cytokines such as TNF-alpha and IL-10, which cause apoptosis, exhaustion, and inhibition of TL proliferation. Not the least, lymphopenia could be the result of redistribution in the lungs and lymphoid organs [81, 84].

In the most severe disease cases, a sudden and rapid clinical deterioration occurs, which is associated with increased levels of acute phase reactants, coagulopathy, and cell lysis, and high proinflammatory cytokine levels, suggesting a second wave of cytokines, responsible for the so-called cytokine storm [81].

The triggering factor of the cytokine storm seems to be immunodeficiency caused by the decrease in the number and the dysfunction of T lymphocytes. Although other innate immunity hyperactivation mechanisms are supposed to be responsible, the cytokine storm is much more likely to occur as a result of a delayed response of innate immunity, followed by persistent hypercytokinemia and an abnormal response of the acquired immune system through T lymphocytes. The result is the failure to eliminate apoptotic cells or macrophages migrated to the site of inflammation and continuous antigenic stimulation by failure of viral clearance. These cells will continue to secrete proinflammatory cytokines, of which the most important are IL-18 and IFN-*γ*, which restimulate macrophage activation. Thus, a vicious circle is created which culminates in cytokine secretion, hemophagocytosis, coagulopathy, and ARDS [82, 85].

### 5.1. Cytokines and the Correlation with the Severity of the Disease

The first evidence of this correlation comes from the study conducted by Huang et al. in a sample of 41 patients who had the plasma levels of several cytokines and chemokines measured. The authors observed that the initial plasma levels of IL-1B, IL-1RA, IL-7, IL-8, IL-9, IL-10, FGF, GCSF, GMCSF, IFN-*γ*, IP-10, MCP1, MIP1A, MIP1B, PDGF, TNF-*α*, and VEGF were higher in all COVID-19 patients compared to healthy persons, the plasma concentrations of IL-5, IL-12p70, IL-15, eotaxin, and RANTES were similar in patients infected with SARS-CoV-2 and healthy persons, and the levels of IL-2, IL-7, IL-10, GCSF, IP-10, MCP1, MIP1A, and TNF-*α* were significantly higher in patients with severe forms of the disease requiring intensive therapy compared to those with mild or moderate forms [86]. Since then, many studies have been conducted in the attempt to elucidate the pathogenic mechanisms of the exacerbated immune response associated with SARS-CoV-2 infection and in the attempt to identify laboratory markers that correlate with the severity and prognosis of the disease in order to achieve a stratification of patients for adequate management based on early therapeutic intervention.

A recently published meta-analysis of 50 studies showed statistically significantly higher values of IL-2, IL-2R, IL-4, IL-6, IL-8, IL-10, TNF-*α*, and INF-*γ* in patients with severe forms of the disease compared to the others. In contrast, there were no significant differences between IL-17 and IL-1*β* values. As it can be seen, in some cases, there is an excessive production of proinflammatory as well as anti-inflammatory cytokines (IL-2R, IL-10), which highlights the dual pathogenic mechanism responsible for the occurrence of the cytokine storm [87]. Another meta-analysis and extensive systematic analysis shows that in patients with severe forms of the disease, lymphocytopenia (decreased CD3, CD4, and CD8 T lymphocytes), leukocytosis, high values of ESR, procalcitonin, LDH, and ALT occur more frequently. The levels of inflammatory cytokines, especially IL-6, 8, 10, and 2R and TNF-alpha, were significantly increased [88].

Regarding the profile of leukocytes, both meta-analyses evidenced a significant decrease in CD4 and CD8 T lymphocytes in the group of patients with severe disease forms [87, 88].

The most studied interleukin is perhaps IL-6, given that tocilizumab, a monoclonal antibody directed against the IL-6 receptor, can be used as therapy for COVID-19 patients who present signs of hyperinflammation. Mojtabavi et al. show in their analysis of 11 studies that IL-6 values are significantly higher in patients with severe forms of COVID-19 compared to those with mild or moderate forms [89]. Furthermore, Laguna-Goya et al. elaborated a model for predicting the risk of mortality in hospitalized COVID-19 patients based on IL-6 values. This includes 5 parameters: FiO_2_/SatO_2_ ratio, neutrophil/lymphocyte ratio, IL-6 value, LDH value, and age. This model might help to stratify patients into more uniform groups from a clinical and biological point of view before their inclusion in randomized clinical trials evaluating the efficacy of tocilizumab or other drugs. Until completion of clinical trials, this model could be used to select patients that would benefit the most from immunomodulatory therapy [90].

The prognostic value of IL-6 was also demonstrated in another study, where it was incorporated along with CD8+ TL into a prognostic model. The authors of the study showed that IL − 6 values > 20 pg/mL and CD8 + TL values < 165 cells/*μ*L are correlated with mortality, being a better indicator of in-hospital mortality than the CURB-65 score [91].

Other cytokines were studied in the attempt to identify the prognostic factors of disease severity and prove their usefulness. An example is represented by IL-2R, included in several prognostic models such as the IL-2R/lymphocyte ratio, as demonstrated in the study conducted by Hou et al. [92], or the model developed by another group which incorporates IL-2R, the values of neutrophils, lymphocytes, and thrombocytes [93]. Another study proposes to monitor IP-10 and MCP-3 values early during the course of the disease in order to identify patients at risk for hyperinflammation and implicitly for more severe forms of the disease [94].

## 6. Therapeutic Targets for the Treatment of COVID-19

Numerous therapeutic targets (Figure 3) have been proposed taking into consideration the various mechanisms of action of SARS-CoV-2 on the endothelium. Regarding the key role of oxidative stress, endotheliopathy, and inflammatory mediators in the COVID-19 pathogenesis [8], we will further present the therapies that counteract the SARS-CoV-2-induced disturbances.

### 6.1. Interleukin-6 Inhibitors

As shown above, IL-6 plays an extremely important role in the occurrence and maintenance of the cytokine storm associated with COVID-19 and is correlated with disease severity, and thus it is an important therapeutic target. In addition, the inhibitors of IL-6 or its receptor proved to be effective in the treatment of other similar syndromes such as HLH associated with Still's disease [95] or in the cytokine storm secondary to CAR-T cell therapy [96]. Regarding their use in COVID-19 patients, only data from case-control studies or case reports are currently available. It should be taken into consideration that these studies were extremely heterogeneous, performed on small samples, with divergent results concerning the monitored indicators (e.g., the need for invasive ventilation and the length of hospital stay). With respect to mortality, the majority showed an increase in survival or at least a favorable trend. Currently, many clinical trials are in progress to evaluate the efficacy and safety of using IL-6 inhibitors in this context. Experimental studies have shown that IL-6 can have a dual effect, both facilitating and suppressing viral replication [23], so that the optimal time of administration is another question that these clinical trials should answer [82, 97–100].

Tocilizumab, sarilumab, and siltuximab are Food and Drug Administration- (FDA-) approved IL-6 inhibitors evaluated for the management of patients with COVID-19 who have systemic inflammation. Tocilizumab is a recombinant humanized anti-IL-6 receptor monoclonal antibody that is approved by the FDA for use in patients with rheumatologic disorders and cytokine release syndrome (CRS) induced by chimeric antigen receptor T cell (CAR-T cell) therapy. Tocilizumab in combination with dexamethasone are indicated in certain hospitalized patients who are exhibiting rapid respiratory decompensation due to COVID-19 [101]. Further findings from REMAP-CAP and the RECOVERY study justify the use of tocilizumab in certain hospitalized patients with rapid respiratory decompensation due to COVID-19 [102].

Sarilumab is a recombinant humanized anti-IL-6 receptor monoclonal antibody that is approved by the FDA for use in patients with rheumatoid arthritis. It is available as an SQ formulation and is not approved for the treatment of CRS [101]. Preliminary efficacy results from REMAP-CAP for sarilumab were similar to those for tocilizumab. Compared to placebo, sarilumab reduced both mortality and time to ICU discharge, and increased the number of organ support-free days; however, the number of participants who received sarilumab in this trial was relatively small, limiting the conclusions and implications of these findings [102].

Siltuximab is a recombinant human-mouse chimeric monoclonal antibody that binds IL-6 and is approved by the FDA for use in patients with multicentric Castleman's disease. Siltuximab prevents the binding of IL-6 to both soluble and membrane-bound IL-6 receptors, inhibiting IL-6 signaling. Siltuximab is dosed as an IV infusion [103]. There are limited data describing the efficacy of siltuximab in patients with COVID-19 [104].

### 6.2. Interleukin-1 Inhibitors

Anakinra is a recombinant IL-1 receptor antagonist, currently approved in the treatment of a number of autoimmune diseases induced by excessive IL-1 secretion, with the aim of reducing inflammation and complications such as ARDS [105].

Starting from the data obtained from the use of anakinra in other similar syndromes such as secondary HLH or macrophage activation syndrome [105] and taking into consideration the high values of this interleukin reported in persons infected with SARS-CoV-2, it was supposed that IL-1 could be an important target in the management of the cytokine storm associated with SARS-CoV-2 as well. A retrospective study showed a clinical improvement in 72% of COVID-19 and ARDS patients treated with this drug [106]. Several randomized clinical trials that test anakinra in COVID-19 patients are underway.

Aside from anakinra, canakinumab, a high-affinity human monoclonal antibody [101], and rilonacept, a soluble IL-1 trap, represent therapeutic options for IL-1 inhibition [107].

Canakinumab counteracts the activity of IL-1 by blocking the interaction between IL-1*β* and its receptor [108]. The beneficial effect of canakinumab for COVID-19 patients results from the improvement of clinical status and reduction of invasive mechanical ventilation needed in these patients together with a prompt amelioration and maintenance in oxygenation levels [109, 110]. Furthermore, canakinumab ameliorates the prognosis of COVID-19 patients and prevents the clinical degradation by blocking the cytokine storm [110].

### 6.3. Anti-TNF-*α*

TNF-*α* is another cytokine with important inflammatory effects, whose increased serum values were also demonstrated in COVID-19 patients. Opinions diverge on the usefulness of anti-TNF-*α* monoclonal antibodies in this context. Infliximab, adalimumab, etanercept, certolizumab, and golimumab are the 5 most commonly prescribed TNFs inhibitors. On the one hand, TNF-*α* inhibition decreases IL-6 and IL-1 concentrations and reduces capillary permeability [111], and studies on animals have shown that the inhibition of this cytokine confers protection against SARS-CoV-2 infection. On the other hand, studies in which TNF-*α* inhibitors were used in syndromes similar to the cytokine storm have reported divergent results, some of them even demonstrating an aggravation of the disease [112].

### 6.4. Type I IFN

Considering the key role of IFN in antiviral response and its immunomodulatory effect, type I IFN seems to be an important potential therapeutic target. Type I IFN was studied both in vivo and in vitro, as monotherapy or in combination with antiviral drugs, in the treatment of SARS-CoV and MERS-CoV infection. Although interferon treatment was demonstrated to be efficient in vitro and in some studies on animals, in human studies the results were divergent. These results can be explained by the limited number of patients included and the heterogeneity of the studies, by the different inhibition mechanisms of the IFN signaling pathway used by the two viruses, as well as by the difficulty in assessing whether the clinical benefit observed was due to IFN or to the drugs with which it was used as part of combined therapy [113].

Another explanation for these results could be the subtype of IFN used as a therapeutic target. Compared to IFN-*α*, IFN-*β* seems to be a much more potent inhibitor of coronaviruses [114]. The time of administration seems to be an important element. Early administration was associated with favorable results, while late administration was associated with significant adverse reactions without an effect on viral replication [115]. In addition, in vitro studies report viral replication inhibition by administration of prophylactic IFN in the case of SARS-CoV-2, while the same strategy is ineffective in the case of SARS-CoV and MERS-CoV [116–118]. A prospective study conducted in China on a sample of 2944 persons working in the health care system showed that interferon administered as a nasal spray is effective in the prophylaxis of SARS-CoV-2 infection [119].

Starting from the information obtained from previous studies on SARS-CoV and MERS-CoV and from the data regarding the pathology of SARS-CoV-2 infection, a number of clinical trials are in progress to test the efficacy of type I IFN in patients infected with SARS-CoV-2.

### 6.5. Inhibitor of Synthetic Serine Protease

Transmembrane protease serine 2 (TMPRSS2) represents the cornerstone in the SARS-CoV-2 S protein interaction with the endothelial cell [120]. TMPRSS2 is a protease that proved its capacity of preventing the cell invasion by SARS-CoV-2 in vitro [52].

Camostat mesylate, an inhibitor of synthetic serine protease infection, could block SARS-CoV-2 spreading in human tissue [120]. Taking into consideration the desirable effects in COVID-19 patients, TMPRSS2 has been approved for clinical use [52].

### 6.6. Recombinant Human ACE2 Protein (rhACE2)

Taking into consideration that SARS-CoV-2 infection induces the depletion of ACE2 receptors, which contributes to systemic and especially pulmonary inflammation, the hypothesis was advanced that administration of recombinant human ACE2 protein can represent a therapeutic target. The causal mechanisms of immune dysfunction and hyperinflammation are multiple, so that the use of rhACE2 as monotherapy is probably insufficient, as demonstrated in patients infected with SARS-CoV in 2017 [76]. There is currently a clinical trial that studies the therapeutic efficacy of this molecule in COVID-19 patients.

### 6.7. JAK Inhibitors

The activated type I IFN JAK1/TYK2-STAT1/2 intracellular signaling pathway plays an important role in cytokine production, so that its inhibition might have a therapeutic effect in the cytokine storm associated with SARS-CoV-2.

Baricitinib is an inhibitor of JAK kinase currently used in the treatment of rheumatoid arthritis, which by selective and reversible binding to JAK receptors disrupts the transduction of the intracellular signal mediated by cytokines and thus attenuates the inflammatory response [121]. In addition, this compound is supposed to inhibit AAK1 receptor, required for viral endocytosis, also inhibiting in this way the entrance of the virus into the host cell [122].

At present, there are several ongoing clinical trials that investigate the efficacy of different JAK inhibitors in COVID-19 patients. An important aspect should be taken into account: the fact that SARS-CoV-2 infection predisposes to coagulopathy and formation of thrombi, and treatment with JAK inhibitors has been associated with an increase in thromboembolic risk [123].

### 6.8. Nitric Oxide

Inhaled nitric oxide (NO) proved its antiviral effects against various coronavirus strains together with the pulmonary vasodilation activity. Of great interest is the ability of NO in the prevention of the development of severe forms of the disease, if administrated at the proper time, at the early stage of COVID-19 [101].

### 6.9. Iloprost

The prostacyclin (PGI2) analogue, iloprost, showed beneficial effects in COVID-19 patients. Iloprost might represent a valuable therapeutic option for respiratory performance improvement [124]. Synthesized in the vascular endothelium, PGI2 plays a role not only in the endothelial barrier homeostasis and platelet aggregation, but it also has anti-inflammatory and vasodilatory effects. [125, 126].

In COVID-19 patients, iloprost could prevent the associated thrombotic events through its protective effects on the endothelium and the antithrombotic activity [124].

### 6.10. The Glycosaminoglycans

Another valuable therapeutic approach is represented by the glycosaminoglycans (GAGs), taking into consideration the double role they play in COVID-19 pathogenesis, their interaction with the chemokines, and the SARS-CoV-2 coreceptor function. Thus, the chemokine interaction with GAGs together with SARS-CoV-2 GAG-mediated cell entry might represent important targets in COVID-19 therapy [127].

### 6.11. Chemokine Receptor 5 Antagonism

The chemokine receptor 5 (CCR5) is a transmembrane structure expressed by several cells, including the endothelial cells [128], and it might be implicated in the SARS-CoV-2 invasion of the endothelial cells. By preventing the SARS-CoV-2 from entering the cell, the CCR5 antagonism could represent a valuable tool in preventing the severe inflammatory response characteristic for COVID-19-associated acute respiratory distress syndrome (ARDS) [127]. CCR5 antagonists proved their efficiency for preventing HIV-1 entry into the cells [129]. Maraviroc, a CCR5 antagonist, blocks the SARS-CoV-2 fusion with other cells (via S protein) and prevents its multiplication [130]. Leronlimab is a monoclonal IgG4 antibody which also has CCR5 as a therapeutic target. Leronlimab successfully reduced the IL-6 levels in patients with severe COVID 19 manifestations [131]. Taking into consideration the role of CCR5 in the COVID-19 pathogenesis and their expression by the endothelial cells, the CCR5 antagonism might represent a therapeutic option in the treatment of SARS-CoV-2-induced endotheliopathy.

### 6.12. The CXCL-8 Pathway

CXCL-8/IL-8 is an inflammatory chemokine that promotes the angiogenesis on endothelial cells via VEGF [132, 133]. The implication of the CXCL-8 pathway in SARS-CoV-2 infection pathogenesis results from its increased circulating levels identified in COVID-19 patients [134]. CXCL-8 is a powerful neutrophil chemotactic factor [135] and its high serum levels in COVID-19 patients might explain the associated neutrophilia. The neutralizing IL-8 antibody therapy and CXCL-8 receptor (CXCR-2) antagonists might represent a therapeutic option for hospitalized COVID-19 patients [127].

## 7. Conclusions

This review summarized the relationship between COVID-19, endothelial dysfunction, inflammation, and oxidative stress. The implication of endothelium in SARS-CoV-2 pathogenesis remains a subject of interest which is intensely researched in current studies. Even though several studies place the endothelial dysfunction and oxidative stress as the main factors responsible for microvascular COVID-19-associated complications, the direct invasion of endothelial cells by SARS-CoV-2 remains disputable. An explanation for the severe COVID-19 manifestations in patients suffering from cardiovascular and metabolic comorbidities might be the endothelial dysfunction associated with the aforementioned conditions; thus, those patients are at high risk for developing pulmonary and extrapulmonary complications. The central role of endothelium in the COVID-19 pathogenesis remains of great interest particularly for its role as a valuable therapeutic target for the prevention and/or treatment of vascular complications in SARS-CoV-2 patients. With a plethora of physiopathological mechanisms, the SARS-CoV-2-induced endotheliopathy appears to play a central role in COVID-19 pathogenesis.

## Figures and Tables

**Figure 1:** Functions of vascular endothelium. Endothelium cells produced some vascular mediators/factors that accomplished the six major functions of normal endothelium (modulation of vascular permeability and vasomotor tone modulation, coagulation homeostasis, inflammation and immunity regulation, cell growth regulation, and oxidation of LDL cholesterol) by which the vascular homeostasis is maintained (adapted after [9]).

**Figure 2:** SARS-CoV-2 enters the human body by binding to ACE2. Activation of RAAS produced a cytokine storm, resulting in the secretion of proinflammatory cytokines/chemokines such as interleukins (ILs), interferon-gamma (IFN-*γ*), monocyte chemoattractant protein-1 (MCP1), and tumor necrosis factor-alpha (TNF-*α*). This storm produces a pleiades of phenomena which is associated with preexistent comorbidities that lead to an increase in disease severity (adapted after [31]).

**Figure 3:** Mechanisms of endothelial dysfunction, inflammation, oxidative stress, and therapeutic targets in SARS-CoV-2 infection. SARS-CoV-2 infection begins when its peak proteins are proteolytically prepared by TMPRSS2, allowing them to bind to ACE2 and initiate viral endocytosis in the EC. This increases the amount of binding of Ang II to AT1R, which in turn activates NADPH-oxidase and subsequently induces an increased production of ROS. These excess ROS mediate signaling pathways that increase the production of inflammatory cytokines (such as IL-1*β*, IL-6, and TNF), decrease the bioavailability of NO and PGI2, and induce endothelial cell apoptosis, leading to endothelial damage and dysfunction. Furthermore, the release of proinflammatory and prothrombotic factors can lead to vascular inflammation, platelet aggregation, and thrombosis. These interactions increase the risk of thrombosis and lung damage in people infected with SARS-CoV-2. ROS also induce an overflow of NETs. There may be several positive feedback loops between cytokines (TNF-*α*, IL-1*β*) and ROS production as well as between cytokines (TNF-*α*, IL-1*β*) and NET formation. ROS, NETs, and proteolytic enzymes released by activated neutrophils also contribute to organ damage and clotting in vessels. Therapeutic targets address SARS-CoV-2-induced feedback loops in EC. Although there have been many therapies proposed to stop the spread of the coronavirus pandemic, those described here address feedback loops involving endothelial dysfunction, oxidative stress, and inflammation. TMPRSS2: transmembrane protease, serine 2; ACE2: angiotensin-converting enzyme 2; AT1R: angiotensin type 1 receptor; ROS: reactive oxygen species; c-Src: protooncogene tyrosine-protein kinase Src; PKC: protein kinase C; IL: interleukin; TNF: tissue necrosis factor; NO: nitric oxide; PGI2: prostaglandin I2 (also known as prostacyclin).
